# Automatic structural scene digitalization

**DOI:** 10.1371/journal.pone.0187513

**Published:** 2017-11-17

**Authors:** Rui Tang, Yuhan Wang, Darren Cosker, Wenbin Li

**Affiliations:** 1 Kujiale.com, Hangzhou, Zhejiang, China; 2 Centre for the Analysis of Motion, Entertainment Research and Applications, University of Bath, Bath, Somerset, United Kingdom; 3 Department of Computing, Imperial College London, London, United Kingdom; University College London, UNITED KINGDOM

## Abstract

In this paper, we present an automatic system for the analysis and labeling of structural scenes, floor plan drawings in Computer-aided Design (CAD) format. The proposed system applies a fusion strategy to detect and recognize various components of CAD floor plans, such as walls, doors, windows and other ambiguous assets. Technically, a general rule-based filter parsing method is fist adopted to extract effective information from the original floor plan. Then, an image-processing based recovery method is employed to correct information extracted in the first step. Our proposed method is fully automatic and real-time. Such analysis system provides high accuracy and is also evaluated on a public website that, on average, archives more than ten thousands effective uses per day and reaches a relatively high satisfaction rate.

## 1 Introduction

CAD floor plans [1] comprise a set of architectural drawings that describe the layout of various structural objects (e.g. walls, windows, doors and furniture) in a building.

In architecture and building design, floor plans contain various levels of detail and show the relationships among rooms, spaces and other architecture components for each level of a structure.

Floor plan analysis can be considered a special image analysis method that attempts to understand the structural and semantic information of a building by analysing 2D versions (Here, ‘images’ refers to both rasterised and vectorised images). After reviewing previous research, it is clear that there are various purposes for analysing a given floor plan. For example, several studies have applied floor plan analysis to the generation of 3D models [2], [3], [4], and another study emphasised interpreting floor plans as CAD formats. In addition, other studies have attempted to detect rooms in architectural drawings [5], [6] and have also searched massive floor plans [7].

[8] is similar to [9] in that they both proposed a method to understand hand-drawn floor plans. In addition, a previous study proposed a complete system for architectural diagram analysis [10], where basic primitives are recognised by applying numerous automated graphics-recognition processes. A method to detect rooms in architectural floor plan images has also been proposed [5]. That method was then adopted and expanded [11] to include new processing steps, such as wall edge extraction and boundary detection.

This paper presents an automatic system for analysing floor plan drawings in CAD format. The remainder of this paper is organised as follows. Work related to this paper is summarised in Section 2. Section 3 provides an overview of the proposed method, including its specific processing steps. Section 4 presents an evaluation of the proposed analysis method and discusses experimental results. Finally, Section 5 concludes this paper and offers suggestions for future work.

## 2 Related work

Architectural drawings, typically in the form of floor plans, are necessary to design, describe and execute a construction project. The architectural elements on each building level are represented using standard symbols and floor plans typically create a top-down orthographic projection.

Floor plans consist of various levels of detailed architectural elements. For example, construction structure drawings (CSD), which are one of the most complicated types of floor plan, portray internal steel bars, the concrete structure of columns, beams, WA walls as well as pipe and ductwork layouts. These drawings are popular with both design engineers and construction managers. Tong Lu and his research team [3] introduced a system that constructs a detailed building model from computer-drawn CSDs. However, interpreting raster images of CSDs requires further research.

Despite floor plans being widely used in architecture engineering and the construction life-cycle as they are able to cover a building’s complete layout, both hand-drawn and computer-produced forms often lack detailed construction information.

Another main drawback arises from the various graphical symbols used in floor plans. Fig 1 shows several common graphical symbols for walls, windows and doors. Note that not all floor plan drawings comply with specific standards. However, the overall purpose of floor plan drawings determines which ones and how components will be shown. Despite the fact that less detailed floor plans can be considered legitimate input by many systems, the various symbols create a challenge when analysing and interpreting floor plan drawings, especially for shape analysis or shape matching methods.

**Fig 1:** Different ways to draw a wall with a window and a door. The variable graphic symbols pose challenges for automatically recognition of objects in CAD drawings [12].

### 2.1 Converting floor plan CAD files

Systems that apply CAD-based floor plans focus more on 3D model extrusion rather than image processing and pattern recognition. Rick Lewis and Carlo Sequin [13] at the University of California, Berkeley, introduced a system that creates 3D polygonal building models semi-automatically by grouping architectural symbols into specified layers in standard DXF files. Their system introduced a correction strategy on disjointed and overlapping edges in order to overcome geometric flaws. This system collects the topology of spaces and portals to generate proper polygon orientation. After each floor is modelled, the system stacks the floors to create a complete model. This system significantly simplifies the recognition process, which benefits designers in various applications, such as smoke propagation simulations.

Clifford So [14] and his colleagues from the Hong Kong University of Science and Technology (HKUST) considered the model conversion problem in a virtual reality context. They targeted three major tasks, i.e. wall extrusion, object mapping as well as ceiling and floor contraction, after observing model reconstruction via a conventional manual method. The processing time of their method is greatly reduced by incorporating automated approaches for each task in the next step, including automatic wall polygon extrusion, generating and placing customised templates of random orientation and size as well as advancing front triangulation. However, their system has a significant disadvantage, i.e. the input file must contain fully established semantic information and no errors, which means the system requires manual intervention. For example, wall lines must be marked by users, architectural objects must be specified, and objects must be assigned to individual transformation matrices.

Researchers at the Massachusetts Institute of Technology (MIT) [15] automated the construction of a realistic MIT campus model (Building Model Generation project (http://city.csail.mit.edu/bmg). Compared to the Berkeley system [13] and whilst a similar pipeline is employed, an additional process is used to position and orient building models automatically using a map for guidance.

Lu’s research team at the Nanjing University of China proposed a system to construct models from computer-drawn CSDs and vectorised floor plans [3]. Compared to other computer drawing formats, symbol recognition in a vector image is much more difficult, because such images contain unlabelled geometric primitives. Similar to the HKUST project [14], this system differentiates walls from other architectural elements. First, it detects parallel line segment pairs as walls, which are then removed from the drawings. Next, the remaining primitives are recognised by detecting feature matches with predefined patterns that contain a symbol’s graphical primitives and contextual information. In the recognition process, the system places patterns in order relative to their priority and checks each, one by one. Corresponding elements are removed from the drawing as soon as they satisfy all of a given pattern’s constraints. Whilst this does require high-quality input, the system benefits users significantly because it focuses on structural details and is highly automated.

### 2.2 Image parsing and drawing analysis

This process analyses an input raster floor plan image and extracts layout information, which is referred to as a ‘parse process’. Referring to Yin’s survey [12], the challenges in this step are explained in Table 1.

**Table 1:** The challenges of image parsing and drawing analysis.

Step	Issues
**Noise removal**	Notation leading lines can easily be confused with wall lines. The background may contain a grid or decorative pattern.
**Text extraction**	Textfont, size and orientation may vary. Text and graphical symbols may share pixels (overlapping or touching).
**Vectorisation**	Most algorithms recover only lines and arcs. Free-form curves are a challenge. Noise affects the result significantly. Vectorisation may yield poor results at junction points.
**Symbol recognition**	Symbols may not comply with standards. There may be a large pool of symbols, and the differences between two symbols may be subtle.

Graphical document analysis technology is required to analyse and parse image floor plans, which includes two main steps: (1) removing noise, such as text and annotation; and (2) graphical symbol recognition. The cleaning step focuses on removing noise and other irrelevant information to improve image quality. In the graphical symbol recognition step, the system categorises the recognised symbols by identifying certain information, including location, orientation and scale.

Compared to other graphical documents, floor plans have certain distinguishable features. For example, various line shapes (curved or straight) represent walls in floor plans. Another difference is that the architectural symbols are made up of simple geometric primitives. Typically, to handle such input, graphics recognition is integrated with vectorisation.

#### 2.2.1 Noise removal

Sampling noise introduced by digital scanning is very common when processing hand-drawn floor plans. However, they are generated by a computer gradually and thus, noise has a broader definition in this context. For example, pixels without directly useful information are typically considered noise, including annotation leading lines, dimension lines, furniture and hardware symbols. On rare occasions, a decorative pattern in the background can be misidentified.

In Loria’s system [16], a morphological filter is applied as a fine line between noise and useful pixels. This method is based on the assumption that background patterns and dimension leading lines can be differentiated from useful lines, because they have different thicknesses and styles. [4] makes a similar assumption, filtering input and only thick construction lines can be preserved.

#### 2.2.2 Text extraction

A perfect algorithm should be free from text font, size and orientation as well as being efficient and requiring little manual intervention. Geometric shapes mixed with text incur extra burden for separation and extraction tasks. Text research has been developed for several decades, and its results can be categorised into structural-based (focusing on structural differences) and pixel-based algorithms.

#### 2.2.3 Graphic recognition

The text is separated from graphics in the previous step. Graphic recognition is a process whereby pixels are organised and ordered according to the geometrical description of the building’s layout. Typically, architectural drawings comprise two primary types of information, i.e. structural information and local architectural components.

As shown in Table 1, graphic recognition comprises vectorisation and symbol recognition. Walls are preserved as geometric poly-lines for the extrusion step, because they define the building’s spatial structure. From this perspective, all systems introduce vectorisation and deal with geometric elements, rather than performing symbol recognition on pixels directly.

**Vectorisation** This process, which is referred to as raster-to-vector conversion, transfers image pixels to geometric primitives. The most important aspects of each algorithm are efficiency, robustness and accuracy. The workflow of traditional line-drawing vectorisation involves two steps, as shown in the following table.

Note that correcting joint errors is required after each step. In most cases, vectorisation algorithms can find line segments and circular arcs; however, more complex curves remain a challenge for existing algorithms.

In Step 1, three groups of algorithms, i.e. parametric model fitting, contour tracking and skeletonisation [17], are typically used. In parametric model fitting, Hough transform [18] is applied to detect lines; however, this requires significant amounts of memory and lacks universality.

Contour tracking detects the contour of white pixels (rather than black ones) and recognises connected regions as rooms. This method can deal with simple floors; however, it cannot deal with complicated structures, because it is based on the assumption that white spaces are divided by black wall lines in the image.

Thinning-based algorithms for skeletonisation attempt to search for a curve bones’ medial axis by stripping boundary pixels until a one-pixel wide skeleton remains [19]. Here, one disadvantage is that intersections always confuse the results. Another disadvantage is that thinning-based algorithms require significant time to process, because each pixel is visited multiple times. Typical medial-axis-based algorithms include pixel tracking [20] and run-graph-based algorithms [20]. Medial-axis-based algorithms treat a thick line as a solid shape and its medial axis as a skeleton.

In Step 2, point chains are segmented into sets of lines, poly-lines and circular arcs by estimating curvature or polygonal approximation to identify critical points.

Loria’s system introduces a skeletonisation technique and polygonal approximation to complete the vectorisation process [16]. The CUHK system tracks the contour of black pixels rather than white ones, which differs from contour tracking [4].

**Symbol recognition** This is the most important part of graphical document analysis, and the graphic symbol recogniser (GSR) in this process should be efficient and not limited to either context or affine transformation. It should be noted that previous research has proved that several methods work well in specific areas and generate positive results.

GSRs can be classified as vector based (oriented toward structure) and pixel based (oriented toward statistics). Vector-based GSRs process graphical primitives, such as points, line segments, arcs and circles, in vectorised images. This approach checks primitives in groups to identify a symbol using region adjacency graphs [21], graphical-knowledge-guided reasoning [22], constraint networks [21] and deformable templates [23]. Note that good vectorisation is expected with this approach, which is affine invariant.

Other GSRs are pixel based. Such recognisers process raster images without vectorisation. Such methods focus on the statistical features of a symbol’s pixel information. Pixel-based approaches contain plain binary images [24], living projections and shape contexts [25]. Compared to vector-based approaches, pixel-based ones are more accurate, even though their performance is sensitive to scaling and rotation. Su Yang improved a recognition method by merging pixel-based and vector-based approaches [26].

In Loria’s project, a network is applied to identify the features of a vectorised image’s primitives [16]. Then, segments in the vectorised floor plan are distributed throughout the network to find terminal symbols. A similar, but simpler approach, is employed in the CUHK system, in which a series of geometric constraints are considered symbol patterns. With this approach, raster or vector images of a floor plan can be used to improve recognition accuracy [4].

## 3 Floor plan analysis system

The proposed automatic floor plan analysis system targets engineering uses and takes CAD format floor plans, which can be considered a set of vectorised images with unit information, as input.

Fig 2 illustrates the basic workflow of the proposed floor plan analysis system, which is described in detail in the following. As mentioned previously, the proposed system is available online for engineering uses without any restrictions to the drawing style of a floor plan. This means that the proposed system can accept a wide variety of input data. Therefore, standardised parsing is required to normalise input data in the first step. After standardisation, all of the information provided by the floor plans is represented by the most basic elements, i.e. straight lines and arcs. Then, because floor plans represent structural data, such as walls, windows and doors, a general filter is applied to the lines to obtain effective room structure information. Then, in consideration of excessive filtration in the filtering step, an image-processing-based retrieval method is adopted to correct the filtered result. Finally, the proposed is able to system extract windows and doors from the floor plan.

**Fig 2:** Work flow of the floor plan analysis system. Starting with putting in raw data, followed by the process of standardisation, filtering and rasterising correcting. As a result, walls, windows and doors can be detected.

### 3.1 Data standardization

#### 3.1.1 Problem statement

It is difficult to develop a general automatic system for recognising various types of CAD floor plans, because designers and engineers draw them in different ways. The variety of CAD floor plans can be summarised as follows.

1. Different units are adopted in different CAD floor plans. Architecture designers employ different units (e.g. centimetres, inches and millimetres), according to the given project’s requirements or personal preference.
2. Structural objects can comprise various internal forms. For example, as shown in Fig 1, doors and windows can be drawn in different ways [12], and, even in a single CAD floor plan, load bearing walls (filled polygons) differ from normal walls (parallel lines). Such variable graphic symbols pose challenges when attempting to recognise floor plans automatically.
3. Dimensions are varied in CAD floor plans, according to the intended purpose. For example, for architectural purposes, some CAD floor plans are shown in 3D space, while others are shown in 2D space.
4. In most cases, manifold furniture or annotations are applied, which impede recognition of the primary structural components (i.e. walls, windows and doors). In most cases, manifold furniture or annotations are applied, which greatly disturb the recognition of the main structural components (walls, windows and doors).
5. Some CAD drawings may contain several floor plans in a single drawing (Fig 3), with each one in such drawings being independent. Hence, the proposed system must be able to extract and separate the individual plans.

**Fig 3:** An example of multiple floor plans in a single CAD drawing; systematic clustering is employed to classify lines based on Euler distance.

#### 3.1.2 Solutions

A simple data standardisation process is employed to address the variety of input CAD floor plans. The primary purpose of this process is to normalise all the architecture elements in the floor plans as lines. The process is described as follows.

- The first step is to standardise the units. By reading the unit information of the CAD floor plans, the various units are converted to millimetres.
- Regardless of the composition of structural objects (e.g. lines, solids, triangles, multi-lines, poly-lines or blocks), all such objects in the drawing are decomposed into lines, which is the most basic element in all architecture drawings. Simultaneously, arcs are converted to short and continuous lines.
- The proposed system focuses on detecting walls, doors and windows in a 2D CAD floor plan and hence, 3D floor plans are converted into 2D spaces by calculating the normal of the lines.
- Furniture, which is considered a type of structural object, is decomposed into lines (refer to Step b). Regarding annotations, marker lines are converted into straight lines, and text elements are removed.
- At this point, the architectural drawing now comprises straight lines and arcs. Since the input drawings can contain more than one floor plan, systematic clustering of the lines is employed, based on Euler distance. I define the distance between lines by searching the closest link between lines (Fig 3).
- Then, a 5000-mm threshold is applied so as to cluster all the lines to segment multiple floor plans from a single CAD file.

### 3.2 A fusion strategy system for CAD floor plans analysis

Here, I introduce a fusion strategy system for CAD floor plan analysis. Floor plans always contain information that helps an architect express the actual layout of the structural objects, e.g. walls, doors and windows. However, during floor plan analysis, different types of objects must be interpreted at different points in time using specific strategies. Hence, a fusion strategy system is introduced that combines a set of general filters and an image-parsing method to extract walls, windows and doors from a CAD floor plan. In the filtering stage, the aim is to identify as many correct walls in the floor plan as possible. Walls are one of the essential elements in a floor plan, for other architecture components, e.g. doors and windows, are attached to them. A set of filters needs to be designed to extract information about walls from the input data. Then, by rasterising the CAD floor plan, the aim is to restore any walls that were filtered excessively in the image-processing strategy. Based on the wall analysis results, the proposed system seeks to detect windows and doors. Then, an image-processing-based wall restoration system is employed. Finally, a mechanism is used to detect doors and windows based on the detected walls. These processes are explained next.

#### 3.2.1 General filters

Similar to existing work [10] and [4], in this step, the proposed system extracts walls from a floor plan by applying general filters. The filters are built on the assumption that walls are represented by parallel lines in Fig 4. Based on this assumption, the filters search for parallel lines and define them as wall candidates. The workflow of the filters is explained below.

**Fig 4:** Raw data as input of a floor plan. Parallel lines are targeted in the process of filtering, based on the assumption that they represent walls.

**1. Gradient filter** (*pi*/12) The objective of introducing this filter is to find non-vertical and non-horizontal lines, because based on the assumption that walls lie horizontally and vertically in a floor plan, they can be targeted by applying this filter. It should be noted that some designers draw lines at a slight tilt, so the threshold is set to *pi*/12. In Eq (1), *L*_*raw*_ is the raw input line from the CAD floor plan, and *L*_1_ represents filtered lines after applying the gradient filter. Then, the filtered lines are divided into two sets: the horizontal set (*H*_*s*1_) and the vertical set (*V*_*s*1_), as expressed by Eq (2).

$$\begin{array}{c} L_{1}=f_{Gradient_{filter}\left(pi/12\right)}\left(L_{std}\right) \end{array}$$ (1)

$$\begin{array}{c} \left(H_{s1},V_{s1}\right)=f_{splitHV}\left(L_{1}\right) \end{array}$$ (2)

Fig 5 shows the filtered result *L*_1_ after the gradient filter (threshold *pi*/12) is processed, while the orange and blue lines represent the horizontal set *H*_*s*1_ and vertical set *V*_*s*1_, respectively.

**Fig 5:** Production of a gradient filter, with the orange and blue lines representing horizontal filtered lines and vertical set, respectively. (Threshold: *pi*/12.)

**2. Length filter (2mm)** As mentioned in Section 3.1, arcs are converted into short lines; however, this may generate many short lines. In consideration of the negative effects brought by irrelevant short lines, a length filter (Eq (3)) is applied to eliminate interference by them, thus addressing this issue. The threshold of this length filter is set as 2mm in order to get the most accurate results and to improve work efficiency as well.

$$\begin{array}{c} H_{s2}=f_{length_{filter}\left(1mm\right)}\left(H_{s1}\right),V_{s2}=f_{length_{filter}\left(1mm\right)}\left(V_{s1}\right) \end{array}$$ (3)

In Fig 6, the red and blue lines represent the filtering results *H*_*s*2_ and *V*_*s*2_ after the length filter is applied, respectively.

**Fig 6:** Production of a length filter, with the red and blue lines representing the filtering result after it is applied (Threshold: 2*mm*).

**3. Gap-Filling and line merging (1 mm, 1 mm, loop = 5)** In architectural drawings, small gaps or dislocations may be created when designers draw walls. The proposed system employs a gap-filling loop filter and merges close parallel lines to solve this problem. The gap-filling process is aimed at connecting close lines in *H*_*s*2_ and *V*_*s*2_.

In this process, it is key to determine whether such lines are sufficiently close to each other, so the threshold is set to 1 mm. Then, the line-merging process merges lines in *H*_*s*2_ and *V*_*s*2_ are in a specific distance. Similar to the previous stage, a threshold of the same value (1 mm) is employed in this process in order to merge close parallel lines. Fig 7 shows the results obtained after applying the gap-filling and line-merging processes. In Eq (4), *H*_*s*3_ and *V*_*s*3_ are the filtered products of this process. It should be noted that this process is prone to drift errors; however, small errors will be fixed Section 3.2.2.

$$\begin{array}{c} \left(H_{s3},V_{s3}\right)=f_{merge(1mm)}\left(f_{fill(1mm)}\left(H_{s2},V_{s2}\right)\right) \end{array}$$ (4)

**Fig 7:** Production of fill gap and merge lines processing. The gap filling process applies to lines that are within 1mm of each other.

**4. Removing multiple parallel lines** Commonly, sets of close multiple parallel lines in walls with an equal gap size represent windows (Fig 8). This filter converts such multiple parallel lines in *H*_*s*3_ and *V*_*s*3_ into a pair of parallel lines. As shown in Fig 8, if the outer bounds of such multiple parallel lines are connected to wall lines, a line-splitting filter is employed to split such long lines into segmented short lines.

$$\begin{array}{c} \left(H_{s4},V_{s4}\right)=f_{RML_{filter}}\left(H_{s3},V_{s3}\right) \end{array}$$ (5)

**Fig 8:** Multi-parallel lines with same gaps to represent windows. Applying a line split function to split long lines into segmented short lines, because the outer bounds of windows are connected in walls.

In Eq (5), *H*_*s*4_ and *V*_*s*4_ are the line-splitting filters.

After the line-splitting filter is applied, inner lines in the multiple parallel lines structure are removed and such structures must be detected in the floor plan to achieve this. To this end, a multiple parallel lines structure detector for *H*_*s*3_ and *V*_*s*3_ is employed. For example, with *H*_*s*3_, the distance between lines is less than 300 mm and is marked as a benchmark, and lines in this range are placed into a candidate line group. It should be noted that inner lines in the candidate group are removed, if the number of multiple parallel lines is from three to six and the distance between each line is between 10 mm and 100 mm. Fig 9 shows the results obtained after removing such multiple parallel lines.

**Fig 9:** The results after removing multiple-parallel lines. Inner lines in the multiple parallel lines structure are removed after applying a line-splitting filter.

**5. Length filter (90mm)** After removing the multiple-parallel lines, the remaining parallel lines in *H*_*s*4_ and *V*_*s*4_ can be considered as candidate lines for the construction of walls. However, many irrelevant lines that do not contribute to walls can remain in sets *H*_*s*4_ and *V*_*s*4_.

As described in the previous subsection, the proposed system seeks to find as many correct walls as possible; however, some may have been over-filtered. The method used to restore walls is discussed in Section 3.2.2.

Considering that main walls are typically represented by long pairs of parallel lines, a length filter with a threshold of 90 mm is employed to remove short lines that may cause interference. In Eq (6), *H*_*s*5_ and *V*_*s*5_ denote the production of this length filter. Fig 10 shows the results obtained after applying it. The length filter removes many pairs of short parallel lines that construct short walls.

$$\begin{array}{c} \left(H_{s5},V_{s5}\right)=f_{length_{filter}\left(90mm\right)}\left(H_{s4},V_{s4}\right) \end{array}$$ (6)

**Fig 10:** The results after applying the length filter. It removes pairs of short parallel lines (less than 90mm) that contribute to a short wall.

**6. Connectivity filter** In the proposed method, a line connectivity filter is applied relative to wall continuity. First, line connectivity is determined and then, lines that have no connection with any others are removed. Fig 11 shows the results obtained after applying the connectivity filter. In Eq (7), *H*_*s*6_ and *V*_*s*6_ denote the productions of the connectivity filter in the vertical and horizontal directions, respectively.

$$\begin{array}{c} \left(H_{s6},V_{s6}\right)=f_{connectivity_{filter}}\left(H_{s5},V_{s5}\right) \end{array}$$ (7)

**Fig 11:** Production from applying a connectivity filter, which removes irrelevant lines.

**7. Gap-Filling and line merging (90mm, 50mm, loop = 5)** For gaps between doors and long lines generated by placing furniture against walls, a gap-filling and line-merging filter is applied similar to that discussed in Section 3.2.1. In Eq (9), *H*_*s*7_ and *V*_*s*7_ denote the productions of the gap-filling filter and line-merging filter in the vertical and horizontal directions, respectively. The gap filling filter connects lines in *H*_*s*6_ and *V*_*s*6_, if they are sufficiently close.

When this filter is applied to door gaps, the threshold is set to 90 mm, but this is set at 50mm when applying it to line merging. Considering the fact that walls generally are 120mm-240mm in width, setting 50mm as a benchmark will not disturb the results of wall selection.

In Fig 12, *H*_*s*7_ and *V*_*s*7_ are represented by red and blue lines, respectively.

$$\begin{array}{c} \left(H_{s7},V_{s7}\right)=f_{merge(50mm)}\left(f_{fill(90mm)}\left(H_{s6},V_{s6}\right)\right) \end{array}$$ (8)

**Fig 12:** Production of the second fill gap and merge line processing. This is the process of filling gaps between doors and long lines. The red and blue lines represent Hs7 and Vs7 in Eq 4.9, respectively.

**8. Detecting candidate pairs of parallel lines** After the second gap-filling and line-merging filters are applied, candidate pairs of parallel lines that contribute to walls are identified and here, two constraints are introduced. One is that the distance between the lines in *H*_*s*7_ and *V*_*s*7_ should be between 100 mm and 400 mm.

This constraint ensures that walls with width within this range are detected. The other constraint is that the overlapping length between each pair of lines should be greater than 400 mm, because such lines are more likely to form walls. In Eq (9), *H*_*s*8_ and *V*_*s*8_ denote the productions of this step in the vertical and horizontal direction respectively. Fig 13 shows them as red and blue lines, respectively.

$$\begin{array}{c} \left(H_{s8},V_{s8}\right)=f_{pair}\left(H_{s7},V_{s7}\right) \end{array}$$ (9)

**Fig 13:** Identify pairs of parallel lines as candidates. Parallel lines in the vertical and horizontal directions are marked as red and blue, respectively.

**9. Generate walls** In this step, walls are generated from the candidate pairs of parallel lines in *H*_*s*8_ and *V*_*s*8_. Here the, lines between 100 mm and 400 mm from the target line are found and such lines are considered wall candidates. Then, as shown in Fig 14, walls are generated from the overlapping area; however, this method can generate incorrect walls. Hence, such errors have to be fixed in the image-parsing stage (Section 3.2.2).

**Fig 14:** Walls are generated from the candidate pairs of parallel lines; the overlapping areas that marked in yellow are walls.

#### 3.2.2 Image-Parsing wall restoration system

With the above filters, whilst the aim is to extract as many correct walls as possible, the input data are difficult to standardise, which inevitably leads to problems. For example, the proposed system may generate incorrect walls or fail to detect correct ones due to excessive filtering. To address this, a wall restoration method based on image parsing of vectorised CAD floor plans is employed. An image-processing technique is not employed to recognise floor plans in CAD format [3][14], if the vectorised parsing method is applied. However, the proposed system integrates the filtered results with an image-parsing mechanism. With analysis of the rasterised image, this system evaluates the wall candidates generated from the first step. More specifically, first, the CAD floor plan and the filtered results are rasterised. Then, the components in the floor plan image are extracted by applying an image component segmentation method. The wall restoration method is discussed in Section 3.2.2.

**Rasterisation** The proposed method converts CAD format floor plans into images. It should be noted that floor plans must be rasterised before the image-parsing method is applied to the vectorised CAD format floor plans. Thus, a raw CAD floor plan and the detected walls are rasterised as images *I*_*raw*_ and *I*_*walls*_, respectively, at equal image resolution (i.e. 4096x4096 pixels). Fig 15 demonstrates the rasterised results of the raw input data, while Fig 16 shows those for walls extracted in the filter steps.

**Fig 15:** Floor plan must be rasterised before applying the image-parsing method. This figure shows a rasterised result of raw input data.

**Fig 16:** Floor plan must be rasterised before applying the image-parsing method. This figure shows a rasterised result for walls extracted in the filter steps.

**Component segmentation** In floor plans, wall regions can always be clearly distinguished from other objects. Therefore, image segmentation is employed to classify the components in *I*_*raw*_. In addition, *I*_*raw*_ is a binary image and hence, the image segmentation task can be converted into a labelling task for connected components in *I*_*raw*_. A connected component in a binary image is a set of pixels that form a connected group. For example, the binary image (left part of Fig 17) [27] has three connected components. The connected component labelling process identifies these in the binary image and assigns a unique label to each [27] (right part of Fig 17). b. The proposed method employs an eight-connectivity-based two-pass connected component labelling method similar to [28]. The pseudocode of this algorithm is shown in Fig 18. The algorithm makes two passes over the image, with the first assigning temporary labels and records equivalences, whilst the second replaces each temporary label with the smallest label of its equivalent class. The following is performed in the first pass:

1. Each element of the data is iterated by column then by row (raster scanning);
2. If the element is not the background;
  - Get the neighbouring elements of the current element;
  - If there are no neighbours, uniquely label the current element and continue;
  - Otherwise, find the neighbour with the smallest label and assign it to the current element;
  - Store the equivalent between neighbouring labels.

**Fig 17:** Left: An example of connected components in a binary image with three connected components. Right: An example of labelling connected components in a binary image. Connected components in the binary image are identified before being a new unique label.

**Fig 18:** Pseudocode of the connected component labelling algorithm. Temporary equivalent labels are assigned in the first passes and the smallest label of its equivalent class will replace them in the second pass.

The following is performed in the second pass:

1. Iterate through each element of the data by column and then by row;
2. If the element is not the background, relabel it with the lowest equivalent label.

Fig 19 shows component labelling result *I*_*rawComponent*_.

**Fig 19:** After applying the two-pass algorithm over the image, component labelling result *I*_*rawComponent*_ generated.

**Wall restoring** The wall regions in a floor plan are distinct from other objects and hence wall information detected in the filter stage can be matched to labelled components in the original image *I*_*raw*_. By tracking each component in the original image and comparing a single component to a wall mask, the component can be defined as a wall, if more than 40% of the wall region overlaps with the wall mask. Fig 15 shows the result after a raw process of wall restoration.

However, the product of rough wall restored by wall candidate mask still has some outliers compared to the ground truth and hence, in order to optimise the wall mask, two extra constraints are introduced.

The first filter considers the factor that walls have strong connectivity with each other. Hence, in this filter, unattached regions, which are not connected to each other, are detected and removed. More specifically, unattached regions will not be identified as an effective wall, if their area or length and width are less than specific thresholds (in these experiments, the threshold of length and width is 2000mm and 200mm, respectively), and they will be eliminated.

After that, the second constraint takes into account another factor that walls should construct a room. In the real drawing, furniture in the corner that includes a sofa may generate parallel lines as well. Instead of connecting to other lines to generate an independent region, these parallel lines may meet the condition of forming walls. If so, the occupancy rate of the mask is increased to 40% plus, which would be marked as walls. To get around this problem, a limitation needs to be set. If the region takes more than 50% of the rectangle space of that generated by plotting the minimum value and the maximum value on the X and Y axis, there is a tiny possibility of being defined as walls, because these normally do not take up a large area in a CAD drawing. Moreover, in order to avoid interfering the process of detecting small walls, the length and width of the rectangle space are much larger than width of an independent wall. In view of the smallest rooms in the real world, the thresholds are set as 2000mm

Fig 20 shows the final wall extraction result obtained by the proposed system.

**Fig 20:** Wall restoration is the process of tracking each component in the original image and comparing a single one with a wall mask, and this figure shows the final wall extraction result obtained by the proposed system.

#### 3.2.3 Detect windows and doors

**Door detection** Typically, doors are attached to walls, i.e. they do not exist independently and, hence they are identified by detecting arcs that are close to detected walls. Normally, arcs with a 90 degree central angle of radius 300 mm to 25000 mm are considered doors.

**Window detection** Window detection is similar to door detection, because windows and doors are both attached to walls. In the proposed method, windows are detected as a part of a wall (Section 3.2.1). Thus, it is possible to find windows by searching multiple parallel lines that are less than 20 mm apart. Also, if the distance between the central line of a group of multiple parallel lines and that of its corresponding wall is less than one-quarter of the wall thickness, this group of multiple parallel lines is considered as a window.

## 4 Evaluation

It is hard to quantitatively evaluate the CAD extraction system because there is barely proper ground truth publicly available. To give an intuitive sense on precision of our system, we implemented the proposed architectural drawing recognition system using Java; we then deploy the proposed system onto Kujiale.com which is a Chinese leading Internet company in interior design. In this case, The proposed system, which is freely available online, incorporates a mature human-computer interaction and representation system. Users can obtain recognition results by uploading CAD floor plans (DWT or DWG format). Fig 21 shows samples from real customers who actually perform analyzing CAD floor plans for three different real-life projects. Please note that such components extraction is achieved without user intervention.

**Fig 21:** The result of analysing CAD floor plans for three different real-life projects. The evaluation result proves that the system is able to complete recognition process without user intervention.

To evaluate the efficiency of our system, we record the usage of every system call then obtain the time consumption (on a mid-ranked Xeon server). On average, the proposed system requires only 2.3 second to extract information from a CAD floor plan. Compared to Lu’s [3] system, which requires nearly one hour to parse a document with 72000 graphic primitives, the proposed system requires approximately 5 seconds to parse a complicated floor plan with a massive number of objects, e.g. more than 35000 lines. The improved efficiency of the proposed system is primarily due to the high-performance algorithm.

Moreover, as mentioned previously, the proposed system can detect a large proportion of walls in most cases. Because the proposed system is intended for practical application by different types of designers, it is difficult to obtain a ground truth for all floor plans. However, due to the lack of a CAD floor plan database, the proposed system was evaluated in a user study. We asked users to score the recognition results of our system (1 means not satisfied and 10 means very satisfied). As shown in Fig 22, based on the research, we get an average score at 7.71 from 2515 user study samples, which indicates an outstanding performance of the system

**Fig 22:** Based on the research, we get an average score at 7.71 from 2515 user study samples, which indicates an outstanding performance of the system.

Meanwhile, according to the statistic on CAD recognition system, the number of recognition requests fluctuated at 80,000 each week between March and July in 2017. The Fig 23 bottomed at 70,000 on week of 4th April and reached the peak at approximately 98,000 on week of 13th June.

**Fig 23:** Statistic of our CAD recognition System. There are over ten thousands request per day.

## 5 Conclusion and further work

A complete system for automatic detection and labeling of architectural elements from CAD format floor plan drawings has been proposed. The proposed system consists of structural and semantic analysis processes to identify relevant information and filter irrelevant information simultaneously. By applying these processes, useful architectural components, such as walls, windows and doors, can be extracted.

Although the theory behind such systems has frequently been discussed over the last two decades, no mature system has been developed for general use. Before the release of the proposed system, manual processes have dominated the market (AutoCAD Revit [29] and Chief Architect [30]). However, the results of a user evaluation (4500 uses per day) demonstrate that the proposed system is efficient and effective.

In China, the large population and increasing urbanisation have increased the need for new housing, which has stimulated rapid real estate development. In consideration of the proposed system’s contributions, we believe that it can have significant economic influence by benefiting the architectural industry.

Based on previous discussion and evaluation, the system that proposed in this paper outperform previous method by reducing processing time to just 2-3s. Meanwhile, the system achieves an impressive satisfaction rate that nine out of ten of the targeted users are satisfied with the result.

In future, we plan to improve the proposed system in several ways. For example, currently, the proposed system is weak when detecting arc walls. Thus, further research into detecting arcs more efficiently is planned. Another problem is that, if the user defines the unit in a floor plan incorrectly, the proposed system will fail to extract anything from the floor plan. Therefore, this issue must be addressed in future. Furthermore, constructing 3D models from 2D floor plans is required by both designers and scientists; thus, we also plan to address the 3D model construction issue.
